The article "A Study on the Application of Extended Care Based on the Biopsychosocial Medicine Model in People with Abnormal Tumor Markers on Physical Examination" was published in 2022. Journal: Contrast Media Mol Imaging.

# A Study on the Application of Extended Care Based on the Biopsychosocial Medicine Model in People with Abnormal Tumor Markers on Physical Examination

**DOI:** 10.1155/2022/7547001

**Published:** 2022-08-08

**Authors:** Wenting Wang, Chunyu Lin, Hong Yu, Shuai Zhou

**Affiliations:** ^1^Department of Physical Examination, Fenyang Hospital Shanxi Province, Fenyang, China; ^2^Department of Emergency, Qingdao Hospital of Traditional Chinese Medicine (Qingdao Hiser Hospital), Qingdao, China; ^3^Translational Research Institute, Henan Provincial People's Hospital, Zhengzhou, China

## Abstract

The purpose of this study was to explore the value of extended care based on a biopsychosocial medicine model in patients with abnormal tumor markers on physical examination. One hundred and fifty-two cases with abnormal primary screening tumor markers who were examined in our medical examination center between January 2020 and January 2022 were selected as the subjects of this study and divided into intervention and control groups according to the random number table method, with 76 cases in each group. The control group was given the usual extended care intervention and the intervention group was given the extended care intervention based on the biopsychosocial medicine model. The compliance rates of regular follow-up, reasonable diet, appropriate exercise, and regular rest were compared between the two groups. After the intervention, the disease-related knowledge score in the intervention group was higher than that in the control group (*P* < 0.05). The compliance rates of regular return visits, reasonable diet, appropriate exercise, and regular routines in the intervention group were higher than those in the control group (*P* < 0.05). After the intervention, the scores of psychological states such as anxiety, depression, and post-traumatic growth in the intervention group were better than those in the control group (*P* < 0.05). After the intervention, the total scores of objective support, subjective support, support utilization, and social support in the intervention group were higher than those in the control group (*P* < 0.05). After the intervention, the intervention group had higher positive coping scores and lower negative coping scores than the control group (*P* < 0.05). Continuing care based on the biopsychosocial model of medicine is effective in people with abnormal tumor markers on medical screening. It can improve the knowledge about the disease, increase the compliance rate, improve negative emotions, psychological status, and social support, and promote a more positive way of responding.

## 1. Introduction

With the change of modern people's living habits and diet structure, the incidence of malignant tumors is increasing year by year. According to statistics, the number of new cases of malignant tumors in China is as high as 4.57 million and the number of deaths is as high as 3 million, which are ranked the foremost in the world [1]. Monitoring tumor marker levels during regular medical checkups is currently an effective way to prevent and screen for tumors, and in the course of clinical application, some medical checkups can screen positive for tumor markers. However, not all patients have the correct knowledge of the results after the medical report is issued [2]. In addition, the physical examination population lacks timely and effective follow-up and social psychological intervention after leaving the hospital, which makes some physical examination people unbalanced due to abnormal examination results, unable to review or receive treatment on time, resulting in delayed illness [3]. It has been reported that the implementation of extended care interventions can help to increase the follow-up rate of patients with abnormal tumor markers and improve their psychological state [4]. The biopsychosocial model of care intervention is a new approach to care based on a modern medical model that takes into account the physical, psychological, and social factors of the care recipient to provide the care they need [5]. At present, there are few studies on the continuation of the biopsychosocial model of nursing intervention in patients with tumor marker abnormalities in medical checkups. Based on this, this study implemented the continuation of the biopsychosocial model of nursing care in patients with tumor marker abnormalities admitted to our medical checkup center in the past two years to observe its application effect.

The article "A Study on the Application of Extended Care Based on the Biopsychosocial Medicine Model in People with Abnormal Tumor Markers on Physical Examination" was published in 2022. Journal: Contrast Media Mol Imaging.

## 2. Patients and Methods

### 2.1. Patients

152 patients with abnormal tumor markers who were admitted to our physical examination center from January 2020 to January 2022 were selected as the subjects of this study and divided into the intervention group and control group according to the random number table, with 76 cases in each group. There was no significant statistical difference (*P* > 0.05) between the two groups in terms of gender, age, education, and other general data, which were comparable (Table 1). This study was approved by the Ethics Committee of Fenyang Hospital Shanxi Province. Signed written informed consents were obtained from all participants before the study.

The inclusion criteria was as follows: (1) all of them were found to be positive for serum carcinoembryonic antigen, alpha-fetoprotein, glycoprotein antigen, and other tumor markers for the first time; (2) patients aged 18 to 75 years old; (3) the clinical data were complete, informed, and agreed to this study. The exclusion criteria was as follows: (1) patients who had been diagnosed with malignant tumor; (2) patients with blood system diseases, autoimmune diseases, or acute and chronic infectious diseases; (3) patients with mental disorders, unable to communicate normally, and difficult to understand the contents of care; (4) patients who could not cooperate to complete this follow-up.

### 2.2. Methods

In the control group, routine continuity of care services were given, physical examination reports were provided to the examinee, the examinee was suggested to maintain a scientific diet and lifestyle habits, and the examinee was advised to come to the hospital on time for follow-up examinations, and was informed of the time, items, and significance of the follow-up examinations. In the intervention group, continuing care interventions based on the biopsychosocial model were as follows: (1) establishment of a continuing care intervention team based on the biopsychosocial model. 4 highly qualified nurses form the intervention team and are trained in the biopsychosocial model before providing care. A health profile was created, taking into account the patient's own situation, and a continuity of care intervention plan based on the biopsychosocial model was developed. (2) Follow-up: team members used telephone, WeChat, and family visits to follow-up with patients who had abnormal tumor markers. During the follow-up visits, they repeatedly provided health education to the patients, informing them about the test results, precautions, and the role of retesting. The pathology information was collated into a personal health file and centrally fed back to the doctor. At the same time, during the follow-up visit, the team should understand the health checker's living habits, work and rest patterns, and dietary preferences, and suggested that the health checker should correct any unreasonable points, so as to maintain a reasonable diet, work and rest, and sleep, and develop healthy living habits. (3) Emotional support: the team should establish good communication and trust with the patient through several follow-up visits, listen to the patient's true thoughts and feelings, grasp the patient's emotional and psychological state, help the patient establish a correct view of tumor marker testing, eliminate the patient's tension and fear of abnormal results, help the patient relieve anxiety and depression and other psychological burdens, and calm the patient's emotions. Appropriately, the team should also help the patients to relieve their anxiety, depression, and other psychological burdens, reassure their emotions, tell them about successful and warning cases, inform them of the importance of early screening, encourage them to come to the hospital for follow-up examinations on time in order to exclude or confirm the diagnosis of tumors at an early stage, and help them to build up their confidence by giving them sufficient emotional support and to meet the follow-up examinations with a positive attitude. (4) Guidance on follow-up examinations: members of the intervention team helped those who had previously been followed up to make appointments for follow-up examinations, and reminded them again by phone one day before the follow-up examination time. The reminders included precautions before the follow-up examination, the procedure of the follow-up examination, the contents of the follow-up examination, and the time of the follow-up examination, to ensure that the examinee completed the follow-up examination smoothly and to avoid other factors interfering with the results. Physical examinees in both groups continued to intervene for 45 days.

The article "A Study on the Application of Extended Care Based on the Biopsychosocial Medicine Model in People with Abnormal Tumor Markers on Physical Examination" was published in 2022. Journal: Contrast Media Mol Imaging.

### 2.3. Observation Index

Disease-related knowledge: a self-made questionnaire on disease-related knowledge was developed with reference to the literature [6], which contained the significance of tumor marker detection, the significance of positive results, examination precautions, the significance of return visit, and the importance of return visit, etc., with a total score of 100 points, indicating that the physical examinees had a better disease-related cognition level. Compliance behavior [7]: after the intervention, the compliance behavior such as regular return visit, reasonable diet, appropriate exercise, and regular routines of the two groups of physical examinees were evaluated, respectively, and the evaluation dimensions were complete compliance, partial compliance, and complete noncompliance, those who met complete and partial compliance were regarded as compliance, and those who met complete noncompliance were regarded as noncompliance, and the compliance rate of the two groups of physical examinees was compared. Psychological state: before and after the intervention, the mental state of the two groups of physical examination subjects was evaluated using the Hospital Anxiety and Depression (HAD) Scale [8] and the Chinese version of the Chinese-Posttraumatic Growth Inventory (C-PTGI) [9]. The HAD scale contains two parts: anxiety subscale and depression subscale, with 7 items in each suitable. The total score is 9 points, 0∼8 points without anxiety and depression symptoms, 9∼21 points with anxiety and depression symptoms, representing more severe degree of anxiety and depression of the physical examination subjects. There are a total of 20 C-PTGI scales, including five dimensions: life perception, personal strength, new possibility, relationship with others, and self-transformation. A six-level scoring system of 0, 1, 2, 3, 4, and 5 is used, with a total score of 100 points, representing more physical examinee grows after trauma. Social support: before and after the intervention, the social support rating scale (SSRS) [10] was used to evaluate the social support of the subjects in the two groups. The SSRS scale had 10 items, including three parts: objective support (2, 6, 7 items), subjective support (1, 3, 4, 5 items), and social support utilization (8, 9, 10 items). The items 1–5 and 8–10 were scored with 1, 2, 3, and 4 items. The items 6 and 7 were scored as 0 point for “no source.” There were several sources to count. The total score was the sum of the scores of each part. The score represented that the social support of the subjects was better. Coping style: before and after the intervention, the trait coping style questionnaire (TCSQ) [11] was used to evaluate the coping status of the physical examinees in the two groups, with a total of 20 items of TCSQ questionnaire, including two major parts: positive coping and negative coping. The five-level scoring system was used. A higher positive response score means that the examinee was more positive and a higher negative response score means that the examinee was more negative.

The article "A Study on the Application of Extended Care Based on the Biopsychosocial Medicine Model in People with Abnormal Tumor Markers on Physical Examination" was published in 2022. Journal: Contrast Media Mol Imaging.

### 2.4. Statistical Analysis

The Statistical Product and Service Solutions (SPSS) 22.0 software (IBM, Armonk, NY, USA) was applied for processing and analysis. Measurement data were expressed as ($\bar{x}$ ± *s*) by using the *t*-test, and the count data were expressed as percentages by using the chi-square test. *P* < 0.05 was considered a statistically significant difference.

## 3. Results

### 3.1. Disease-Related Knowledge Scores between the Two Groups

There was no significant difference in disease-related knowledge scores between the two groups before intervention (*P* > 0.05), and the scores in the intervention group were higher than those in the control group after intervention (*P* < 0.05), as shown in Table 2.

### 3.2. Compliance Behavior between the Two Groups

The compliance rates of physical examinees in the intervention group such as regular return visits, reasonable diet, appropriate exercise, and regular routines were higher than those in the control group (*P* < 0.05) (Table 3).

### 3.3. Psychological Status between the Two Groups

There was no significant difference in the scores of psychological status such as anxiety, depression, and post-traumatic growth between the two groups before intervention (*P* > 0.05), and the scores of psychological status such as anxiety, depression, and post-traumatic growth in the intervention group were better than those in the control group after intervention (*P* < 0.05) (Table 4).

The article "A Study on the Application of Extended Care Based on the Biopsychosocial Medicine Model in People with Abnormal Tumor Markers on Physical Examination" was published in 2022. Journal: Contrast Media Mol Imaging.

### 3.4. Social Support between the Two Groups

There was no significant difference in objective support, subjective support, support utilization, and total social support score between the two groups before the intervention (*P* > 0.05), and the objective support, subjective support, support utilization, and total social support score in the intervention group were higher than those in the control group after the intervention (*P* < 0.05) (Table 5).

### 3.5. Coping Style Scores between the Two Groups

There was no significant difference in positive coping and negative coping scores between the two groups before the intervention (*P* > 0.05), and the positive coping score of the intervention group was higher than that of the control group and the negative coping score was lower than that of the control group after the intervention (*P* < 0.05) (Table 6).

## 4. Discussion

With the rapid increase in the incidence of malignant tumors in recent years, tumor marker tests such as carcinoembryonic antigen, alpha-fetoprotein, and glycoprotein antigen have become a routine part of medical check-ups for residents, and are important for the early detection and treatment of malignant tumours [12]. When the examination results of tumor markers are abnormal, it suggests the possibility of cancer, and timely and effective return visit is required to further rule out or diagnose cancer.

However, in actual clinical practice, some medical examiners may lack knowledge about the disease, resulting in anxiety, depression, and panic, and thus avoiding follow-up consultations [13], and the lack of effective extended care interventions in hospitals may delay the condition and cause the examiners to miss the best time for treatment, which is not conducive to personal, family, and social harmony and stability [14].

In this study, routine continuous nursing was used as a control, and continuous nursing based on biopsychosocial medical model was used to provide nursing services for physical examination patients in the intervention group. The results showed that the compliance rate of disease-related knowledge score, regular return visit, reasonable diet, appropriate exercise, and regular routines of physical examination patients in the intervention group was higher than that in the control group (*P* < 0.05), indicating that continuous nursing based on biopsychosocial medical model could improve disease-related knowledge and compliance behavior of patients with abnormal tumor markers in physical examination, promote their return visit on time, and maintain healthy living habits. Those with abnormal tumor markers in physical examination do not understand the meaning of test results due to their lack of understanding of disease-related knowledge, or excessively interpret test results, resulting in significant changes in their psychological status, easy self-abandonment, and development of bad living habits and dietary habits, and some physical examinees may also experience insomnia due to negative emotional distress [15, 16]. Continuing nursing based on the biopsychosocial medical model ensures that the physical examinees fully understand and master disease-related knowledge by establishing a nursing group, strengthening the communication between the group members and the physical examinees, and conducting health education one-on-one to the physical examinees, so that they can better cooperate to adjust bad living habits and go to the hospital for return visits in a timely manner [17]. Therefore, physical examinees in the intervention group had higher disease-related knowledge scores and compliance rates than those in the normal group.

The article "A Study on the Application of Extended Care Based on the Biopsychosocial Medicine Model in People with Abnormal Tumor Markers on Physical Examination" was published in 2022. Journal: Contrast Media Mol Imaging.

The results of this study also found that the intervention group was superior to the control group in the scores of psychological states such as anxiety, depression, and post-traumatic growth (*P* < 0.05), and the intervention group had higher objective support, subjective support, support utilization, and total score of social support compared with the control group (*P* < 0.05). After the intervention, the intervention group had higher positive coping scores and lower negative coping scores than the control group (*P* < 0.05). It is shown that continuous care based on the biopsychosocial medical model can effectively eliminate negative emotions of physical examinees, improve social support, and help them face return visits in an active coping style. When physical examinees get abnormal results, their emotions are greatly affected due to their lack of relevant knowledge, and most physical examinees may experience adverse psychological states such as depressed mood, anxiety, and depression [18]; have a negative attitude towards return visits; and are difficult to actively cooperate to complete further examinations [19]. The members of the continuous nursing group based on the biopsychosocial medical model establish one-on-one communication with the physical examinees by telephone follow-up, follow-up, and family visit to improve the disease cognition of the physical examinees while more clearly understanding the mental stress and worry points they face. The members of the nursing intervention group give psychological counseling according to the physical examinees' own conditions [20], improve social support and their own confidence with the help of their families, encourage the physical examinees to face return visits and possible treatment with a positive attitude, promote their post-traumatic growth, and improve their psychological status as a whole [21]. This article still has several limitations. For example, this study was only conducted on patients with positive tumor markers, and patients diagnosed at a later stage were not followed up again. Besides, the sample size included in this study was small and this study was a single-center study.

The article "A Study on the Application of Extended Care Based on the Biopsychosocial Medicine Model in People with Abnormal Tumor Markers on Physical Examination" was published in 2022. Journal: Contrast Media Mol Imaging.

## 5. Conclusion

In summary, the application effect of continuous nursing based on biopsychosocial medical model in patients with abnormal tumor markers in physical examination is significant, which can effectively enhance the disease-related knowledge of physical examination patients, improve the compliance rate, eliminate negative emotions, improve psychological status and social support, and promote them to establish a positive coping style.

## Figures and Tables

**Table 1:** Baseline data in the study.

Group	*n*	Gender		Age (years)	Educational level			
		Male	Female		Primary school	Junior high school	Technical secondary school and high school	College and above
Intervention group	76	45	31	52.84 ± 5.13	10	25	29	12
Control group	76	44	32	52.77 ± 5.09	9	24	32	11

*t*/*X*^2^		0.027		0.0844	0.264			
*P* value		0.869		0.932	0.966			

**Table 2:** Comparison of disease-related knowledge scores between the two groups ($\bar{x}$ ± *s*).

Group	Preintervention	Post intervention	*t*	*P* value
Intervention group (*n* = 76)	61.34 ± 5.79	85.47 ± 6.76	23.634	<0.001
Control (*n* = 76)	62.05 ± 5.43	78.63 ± 7.18	16.056	<0.001
*t*	0.780	6.047		
*P* value	0.437	<0.001		

**Table 3:** Comparison of compliance behavior between the two groups (*n*, %).

Group	Regular return visit			Reasonable diet			Proper exercise			Regular routines		
	Medical compliance	Noncompliance	Compliance rate	Medical compliance	Noncompliance	Compliance rate	Medical compliance	Noncompliance	Compliance rate	Medical compliance	Noncompliance	Compliance rate
Intervention group (*n* = 76)	54	22	71.05	59	17	77.63	50	26	65.79	61	15	80.26
Control (*n* = 76)	42	34	55.26	46	30	60.53	37	39	48.68	50	26	65.78

Χ^2^	4.071			5.205			4.543			4.041		
*P* value	0.044			0.023			0.033			0.044		

**Table 4:** Comparison of psychological status between the two groups ($\bar{x}$ ± *s*, min).

Group	Anxious		Depression		Post-traumatic growth	
	Preintervention	Post intervention	Preintervention	Post intervention	Preintervention	Post intervention
Intervention group (*n* = 76)	11.33 ± 2.66	6.45 ± 1.37^*∗*^	12.74 ± 2.12	5.36 ± 1.23^*∗*^	63.75 ± 9.84	88.46 ± 2.97^*∗*^
Control (*n* = 76)	11.39 ± 2.43	8.12 ± 1.59^*∗*^	12.83 ± 2.26	6.71 ± 1.47^*∗*^	64.03 ± 11.02	76.95 ± 3.85^*∗*^
*t*	0.145	6.937	0.253	6.140	0.165	20.636
*P* value	0.885	<0.001	0.801	<0.001	0.869	<0.001

^*∗*^ *P* < 0.05, compared with that before intervention in the same group.

The article "A Study on the Application of Extended Care Based on the Biopsychosocial Medicine Model in People with Abnormal Tumor Markers on Physical Examination" was published in 2022. Journal: Contrast Media Mol Imaging.

**Table 5:** Comparison of social support between the two groups ($\bar{x}$ ± *s*, min).

Group	Objective support		Subjective support		Support utilization		Social support total score	
	Preintervention	Post intervention	Preintervention	Post intervention	Preintervention	Post intervention	Preintervention	Post intervention
Intervention group (*n* = 76)	8.47 ± 1.13	12.63 ± 2.78^*∗*^	19.12 ± 2.04	23.87 ± 3.91^*∗*^	7.35 ± 0.92	9.28 ± 1.12^*∗*^	34.96 ± 4.03	45.79 ± 5.31^*∗*^
Control (*n* = 76)	8.45 ± 0.96	11.79 ± 1.65^*∗*^	19.05 ± 2.31	21.94 ± 4.05^*∗*^	7.39 ± 0.81	8.65 ± 0.93^*∗*^	34.88 ± 3.95	42.36 ± 4.77^*∗*^
*t*	0.118	2.265	0.198	2.989	0.284	3.773	0.124	4.198
*P* value	0.907	0.025	0.843	0.003	0.776	<0.001	0.902	<0.001

^*∗*^ *P* < 0.05, compared with that before intervention in the same group.

**Table 6:** Comparison of coping style scores between the two groups ($\bar{x}$ ± *s*, min).

Group	Active response		Negative coping	
	Preintervention	Post intervention	Preintervention	Post intervention
Intervention group (*n* = 76)	23.09 ± 3.07	31.75 ± 3.91^*∗*^	32.63 ± 4.15	20.41 ± 3.29^*∗*^
Control (*n* = 76)	23.16 ± 3.25	28.94 ± 4.68^*∗*^	32.58 ± 4.23	25.67 ± 2.73^*∗*^
*t*	0.136	4.017	0.074	10.726
*P* value	0.892	<0.001	0.942	<0.001

^*∗*^ *P* < 0.05, compared with that before intervention in the same group.

## Data Availability

The datasets used and analyzed during the current study are available from the corresponding author on reasonable request.

## References

[1] Xia C., Dong X., Li H. (2022). Cancer statistics in China and United States, 2022: profiles, trends, and determinants. *Chinese Medical Journal*.

[2] Malinowski D. P. (2007). Multiple biomarkers in molecular oncology. II. Molecular diagnostics applications in breast cancer management. *Expert Review of Molecular Diagnostics*.

[3] Taube B. A., Taube S. E. (2004). Prognostic and predictive markers in cancer. *Disease Markers*.

[4] Jakobsen D. H., Rud K., Egerod H., Egerod I. (2014). Standardising fast-track surgical nursing care in Denmark. *British Journal of Nursing*.

[5] Ilnitski A. N., Prashchayeu K. I., Sultanova S. S., Liutsko V. V., Gorelik S. G. (2019). Bio-psycho-social model of energizing care of the elderly and senile age at home. *Advances in Gerontology*.

The article "A Study on the Application of Extended Care Based on the Biopsychosocial Medicine Model in People with Abnormal Tumor Markers on Physical Examination" was published in 2022. Journal: Contrast Media Mol Imaging.

[6] Silva S., Bártolo A., Santos I. M., Monteiro A., Monteiro S. (2022). Towards a better understanding of the factors associated with distress in elderly cancer patients: a systematic review. *International Journal of Environmental Research and Public Health*.

[7] Dimeo F., Pagonas N., Seibert F., Arndt R., Westhoff W., Westhoff T. H. (2012). Aerobic exercise reduces blood pressure in resistant hypertension. *Hypertension*.

[8] Deng Y., Wang S., Wang J. (2021). Validation of the hospital anxiety and depression scale and the perceived stress scale and psychological features in patients with periodontitis. *Journal of Periodontology*.

[9] Tu P. C., Hsieh D. C., Hsieh H. C. (2020). Positive psychological changes after breast cancer diagnosis and treatment: the role of trait resilience and coping styles. *Journal of Psychosocial Oncology*.

[10] Chen K., Yu S., Zhang Z. (2021). Investigation and analysis of influencing factors of early activity compliance of patients after minimally invasive esophagectomy. *Annals of Palliative Medicine*.

[11] Sisolefsky F., Rana M., Herzberg M., Herzberg P. Y. (2021). Validierung des Düsseldorfer Screeningtools: ein traitbasierter Ansatz zur Erfassung der psychischen Belastung von Krebspatienten. *HNO*.

[12] Thiessen M., Sinclair S., Raffin Bouchal P. A., Raffin Bouchal S. (2020). Information access and use by patients with cancer and their friends and family: development of a grounded theory. *Journal of Medical Internet Research*.

[13] Göral Türkcü S., Özkan S. (2021). The effects of reflexology on anxiety, depression and quality of life in patients with gynecological cancers with reference to Watson’s theory of human caring. *Complementary Therapies in Clinical Practice*.

[14] Yang K., Wu Z., Zhang H. (2022). Glioma targeted therapy: insight into future of molecular approaches. *Molecular Cancer*.

[15] He P., Shen B., Shen S. (2022). Effects of out-of-hospital continuous nursing on postoperative breast cancer patients by medical big data. *Journal of Healthcare Engineering*.

[16] Han D., Wang D., Li J., Li X. (2021). Effect of multidisciplinary collaborative continuous nursing on the psychological state and quality of life of patients with cervical cancer. *American Journal of Tourism Research*.

[17] Gao M., Zhang L., Wang Y. (2021). Influence of humanistic care based on Carolina care model for ovarian cancer patients on postoperative recovery and quality of life. *American Journal of Tourism Research*.

[18] Song P., Huang Q., Huang Y. (2010). Multidisciplinary team and team oncology medicine research and development in China. *Bioscience trends*.

[19] Rojo M. G., Rolón E., Calahorra L. (2008). Implementation of the business process modelling notation (BPMN) in the modelling of anatomic pathology processes. *Diagnostic Pathology*.

The article "A Study on the Application of Extended Care Based on the Biopsychosocial Medicine Model in People with Abnormal Tumor Markers on Physical Examination" was published in 2022. Journal: Contrast Media Mol Imaging.

[20] Morofuji Y., Nakagawa S. (2020). Drug development for central nervous system diseases using in vitro blood-brain barrier models and drug repositioning. *Current Pharmaceutical Design*.

[21] Richmond E. S., Dunn D. (2012). Biomarkers: an overview for oncology nurses. *Seminars in Oncology Nursing*.

